# Predictive Value of Preoperative Dynamic Contrast-Enhanced MRI Imaging Features in Breast Cancer Patients with Postoperative Recurrence Time

This article has been retracted.

**DOI:** 10.1155/2022/9556880

**Published:** 2022-08-02

**Authors:** Zhangqiang Wu, Shaoli Gao, Yefeng Yao, Li Yi, Jianjun Wang, Fei Liu

**Affiliations:** ^1^Department of Surgical Oncology, GuangFu Oncology Hospital, Jinhua 321000, Zhejiang, China; ^2^Department of Geriatrics, The Second Hospital of Jinhua, Jinhua 321000, Zhejiang, China; ^3^Special Inspection Section, Jinhua Wenrong Hospital, Jinhua 321000, Zhejiang, China; ^4^Department of Breast Oncology Surgical, GuangFu Oncology Hospital, Jinhua 321000, Zhejiang, China

## Abstract

Although the implementation of surgery has reduced the mortality of breast cancer, postoperative recurrence is still an important problem bothering patients. DCE-GMRI can not only clearly display the morphological characteristics of breast lesions but also dynamically observe the blood perfusion of the lesions. On account of this, we explored the predictive value of preoperative dynamic contrast-enhanced magnetic resonance imaging (DCE-MRI) imaging features in breast cancer patients on postoperative recurrence time of breast cancer. The results showed that DCE-MRI images can clearly show the hemodynamic characteristics and morphological characteristics of tumor lesions, and have important value in predicting the recurrence time of breast cancer after surgery. The prognosis of early recurrence of breast cancer is worse. DCE-MRI can predict the time of postoperative recurrence and provide important clinical references.

## 1. Introduction

Breast cancer refers to the malignant proliferation of breast epithelial tissue, and is one of the most common malignant tumors in women, which seriously threatens women's health. Breast lumps, nipple discharge, and nipple depression are the main clinical symptoms of breast cancer patients [1]. In recent years, with the development of medical technology, the survival rate of breast cancer patients has greatly improved, but about 40% of patients still experience recurrence after receiving surgical treatment [2]. Therefore, how to predict breast cancer recurrence early and accurately by preoperative noninvasive routine examination is of great significance to reduce the recurrence rate of patients. Common imaging tests for breast cancer include mammography, ultrasound, dynamic contrast-enhanced magnetic resonance imaging (DCE-MRI), etc. DCE-MRI has high soft tissue resolution and can clearly display the hemodynamic characteristics and morphology of tumors. It provides imaging features of tumors for clinical decision-making. Many researchers have predicted the benign and malignant conditions of tumors by extracting the image features in the DCE-MRI of the breast. However, its role in predicting tumor recurrence is still controversial. This article aims to analyze the predictive value of postoperative recurrence time by studying the preoperative DCE-MRI imaging characteristics of breast cancer patients.

## 2. Information and Methods

### 2.1. General Information

The clinical data of 86 patients with postoperative recurrence of breast cancer who were diagnosed and treated in our hospital from May 2012 to May 2015 were retrospectively analyzed. The age ranged from 25 to 75 years old, with an average age of (51.32 ± 9.25) years. According to the recurrence time, 66 patients were divided into the early recurrence group (47 cases) and the late recurrence group (39 cases).

### 2.2. Inclusion Criteria

(1) The diagnosis results were confirmed by postoperative pathology. Conform to the diagnosis of postoperative recurrence of breast cancer in “China Anti-Cancer Association Guidelines and Specifications for Breast Cancer Diagnosis and Treatment” [3]; (2) preoperative breast DCE-MRI examination; (3) the patient had no distant metastasis at the time of diagnosis; (4) recurrence was confirmed after follow-up.

### 2.3. Exclusion Criteria

(1) A history of biopsy, neoadjuvant chemotherapy, or endocrine therapy before DCE-MRI; (2) the pathological stage is T4; (3) male breast cancer.

### 2.4. Research Methods

Philips Ingenia 3.0 T magnetic resonance imaging was used to examine the patient before the operation. During the examination, the patient was kept in a prone position, the breasts were naturally draped, and an 8-channel phased array coil was used for signal acquisition. The patient underwent a conventional triplane localization scan, and the bilateral breast sagittal T2 weighted imaging (T2WI) (with fat suppression) was used for a plain scan. The repetition time/echo time was 4650 ms/85 ms, the slice thickness was 4 mm, the slice spacing was 1.0 mm, the matrix is 320 × 224, the number of excitations is 3, and the field of view is 20 cm × 20 cm. Then, multiphase DCE-MRI was performed with transverse-axis dynamic contrast-enhanced volumetric imaging, and gadopentetate meglumine contrast agent was injected intravenously at a dose of 0.2 mmol/kg and a rate of 3.0 ml/s. After 15∼25 s of contrast agent injection, the 3D FLASH sequence was used for 6 consecutive scans without interruption. The single scan time was 30 s. The parameters were set as follows: repetition time/echo time was 8 ms/3.93 ms, The layer thickness is 0.8 mm, the layer spacing is 0.4 mm, the matrix is 350 × 350, the number of excitations is 0.6, and the field of view is 34 mm × 34 cm. The raw DICOM images of the dynamic enhancement sequence were imported into the Omni-Kinetics software for postprocessing. The reference region model was used, combined with T2WI and DCE-MRI images to determine the location of the lesion, the region of interest (ROI) was manually delineated, the contralateral pectoralis major at the ROI level was selected as the reference, and the hemorrhage in the full pixel area of the tumor lesion was automatically generated by software calculation. Fluid dynamics parameters were measured. DCE-MRI morphological features: select 6-phase dynamic enhanced images under the same scanning parameters and input them into Omni-Kinetics software for morphological feature parameter sphericity measurement.

### 2.5. Observation Indicators

Observation and recording of preoperative DCE-MRI imaging features of breast cancer patients: background parenchymal enhancement (BPE), morphology, lesion edge, intralesional enhancement, increased degree of whole breast blood vessels, adjacent blood vessels of the lesion, and time-signal intensity curve (TIC). DCE-MRI hemodynamic parameters: time to peak (TTP), contrast max concentration (Max Conc), area under the time signal curve (AUC), time signal curve maximum slope (Max Slope), K^trans^, K_ep_, and V_p_. The 6-phase DCE-MRI images and the morphological characteristic parameter sphericity of the same period were compared and analyzed. If it is a true sphere, the result of this parameter is 1. The closer to the sphere, the more regular the lesion, and the closer the value is to 1; otherwise, it deviates from 1 and is less than 1.

Breast cancer recurrence: patients were followed up every 6 months after surgery for more than 5 years. All patients were diagnosed with suspected recurrence by magnetic resonance imaging, bilateral breast ultrasound or bone scan, and confirmed recurrence by biopsy. Postoperative recurrence ≤2 years was regarded as early recurrence, and postoperative recurrence >2 years was regarded as late recurrence.

### 2.6. Statistical Methods

The SPSS 22.0 software was used to process the data analysis, and the measurement data of the experimental data were presented as mean ± standard deviation ($\bar{x}\pm S$), and enumeration data were presented as %. Pairwise comparison of measurement data between groups was analyzed by *t*-test. Differences between groups were compared by the *χ*^*2*^ test. The receiver operating characteristic curve (ROC) was drawn, and the area under the ROC curve was used to evaluate the prediction of DCE-MRI on postoperative recurrence time in breast cancer patients. Kaplan–Meier survival curves were used to analyze the prognosis and survival curves of breast cancer patients with recurrence in different periods, and the log-rank test was used for comparison. *P* < 0.05 indicates a statistically significant difference.

## 3. Results

### 3.1. Comparison of DCE-MRI Features of Breast Cancer Recurrence between Two Groups

There were no significant differences in BPE, morphology, lesion margin, intralesional enhancement, and TIC between the two groups of breast cancer recurrence in DCE-MRI (*P* < 0.05). The increase of severe whole breast blood vessels and the proportion of adjacent blood vessels in the early recurrence group were higher than those in the late recurrence group, and the differences were statistically significant (*P* < 0.05), as shown in Table 1.

### 3.2. Comparison of Breast Cancer Recurrence and DCE-MRI Hemodynamics between the Two Groups

There was no significant difference in TTP, K^trans^, K_ep_ and V_p_ values in DCE-MRI hemodynamics between the two groups (*P* < 0.05). The values of Max Conc, AUC, and Max Slope in the early recurrence group were higher than those in the late recurrence group, and the differences were statistically significant (*P* < 0.05), as shown in Table 2.

### 3.3. Relationship between Breast Cancer Recurrence and DCE-MRI Morphological Features

Comparative analysis of the morphological characteristics of the 6-stage DCE-MRI images showed that in the 3-stage morphological characteristic parameter sphericity, the median of the early recurrence group was 0.06 (0.04, 0.11), which was lower than the median of 0.09 (0.06, 0.12) of the late recurrence group. That is, the tumor shape in the early recurrence group was more irregular, and the difference was statistically significant *P* < 0.05 (*P* < 0.05), as shown in Figure 1 and Figure 2.

### 3.4. The Predictive Value of DCE-MRI for Breast Cancer Recurrence

The area under the curve of DCE-MRI predictive value for time to recurrence after breast cancer surgery was 0.918 (95% CI 0.853–0.983), which was higher than the increase in whole milk vessels, adjacent vessels of the lesion, Max Conc, AUC, Max Slope, and the sphericity of stage 3 morphological characteristic parameters. Moreover, when the optimal cutoff value was 0.710, the sensitivity and specificity of DCE-MRI in diagnosing the postoperative recurrence time of breast cancer were 78.1% and 92.9%, respectively, as shown in Table 3 and Figure 3.

### 3.5. Prognosis of Breast Cancer Patients with Recurrence in Different Periods

As of May 31, 2020, 13 of 86 breast cancer patients died. Among them, the mortality rate of the early recurrence group was 23.40% (11/47), which was higher than 5.13% (2/39) of the late recurrence group, and the difference was statistically significant (*P* < 0.05). The median survival time of the early recurrence group was 26.8 months, which was lower than that of the late recurrence group of 54.3 months. Log-rank test *P*=0.012, the difference was statistically significant, as shown in Figure 4.

## 4. Discussions

Breast cancer is one of the most common malignant tumors in women, with a high incidence rate. In recent years, the incidence of breast cancer in the world is still increasing. Although treatment strategies such as surgery have significantly improved the overall prognosis of patients with breast cancer, a significant proportion of patients develop local recurrence or distant metastasis after treatment Therefore, how to accurately predict the postoperative recurrence of breast cancer and guide clinical treatment is extremely important. Tumor recurrence is related to factors such as vascular distribution and vascular permeability around the tumor. The morphological and hemodynamic characteristics of DCE-MRI can reflect the shape and size of the tumor, the distribution of blood vessels around the tumor, and the degree of vascular permeability. Effective imaging tests for cancer [4]. Therefore, we speculate that it is also effective in predicting tumor recurrence.

The results of this study showed that there was no significant difference in BPE, morphology, lesion margin, intralesional enhancement, and TIC between the two groups of breast cancer recurrence DCE-MRI (*P* > 0.05). The increase of severe whole breast blood vessels and the proportion of adjacent blood vessels in the early recurrence group were higher than those in the late recurrence group (*P* < 0.05). The reason is that the recurrence of the tumor is closely related to the abundant blood supply. The severe increase of blood vessels in the whole breast and the blood vessels adjacent to the lesion can provide abundant blood for the recurrence of breast cancer. The more it is, the easier it is for breast cancer to recur early [5]. There was no significant difference in TTP, K^trans^, K_ep_ and V_p_ values in DCE-MRI hemodynamics between the two groups (*P* > 0.05). The values of Max Conc, AUC, and Max Slope in the early recurrence group were higher than those in the late recurrence group (*P* < 0.05). The reason is that tumor recurrence depends on abundant blood supply, and DCE-MRI can display the vascular properties of tumor sites through intravenous injection of contrast agents, so the recurrence time of tumor can be predicted by observing the results of DCE-MRI [6]. The Max Conc value is the maximum concentration of contrast agent in the lesion. The more contrast agent retained in the lesion, the greater the concentration and the greater the Max Conc value, indicating that the blood supply of this part is richer and the earlier recurrence is easier [7]. AUC can indicate the blood perfusion volume of different tissues in a certain period of time during the dynamic enhancement process. The larger the AUC value, the more blood perfusion at this site, and the easier it is for the tumor to relapse early. And the Max Slope value reflects the blood perfusion and capillary permeability of the tissue. The increase of the Max Slope value indicates that the abundant blood flow in this part is easy to nourish the tumor through the blood vessels and promote the early recurrence of the tumor [8]. The values of Max Conc, AUC, and Max Slope in patients with early recurrence were larger than those with late recurrence, indicating that the blood supply of early recurrence tumors was more abundant than that of late recurrence tumors. Comparative analysis of the 6-stage DCE-MRI imaging characteristic parameters, in the 3-stage morphological characteristic parameter sphericity, the median of the early recurrence group was 0.06 (0.04, 0.11), which was lower than the median of 0.09 (0.06, 0.12) of the late recurrence group. That is, the tumor shape of the early recurrence group was more irregular (*P* < 0.05). The tumor heterogeneity in the early recurrence group is stronger, and the tumor is more aggressive, which is not conducive to the prognosis and survival of the patients, which may be related to the richer blood supply of the tumor in the early recurrence group. This shows that through the comparison of DCE-MRI imaging characteristic images and parameters, the heterogeneity and invasiveness of tumors can be intuitively understood [9, 10].

Furthermore, the area under the curve of the predictive value of DCE-MRI for breast cancer recurrence time was 0.918 (95% CI 0.853–0.983). When the optimal cutoff value was 0.710, the sensitivity was 78.1% and the specificity was 92.9%. The reason is that breast cancer is a vascular-dependent malignant tumor. The growth, development and recurrence of tumor tissue require an abundant microvascular network for oxygen supply, and the more irregular the tumor shape and the stronger the heterogeneity, the easier it is to relapse early. Preoperative DCE-MRI can predict the recurrence time of breast cancer after surgery, and prompt clinicians to prevent and treat in time, thereby improving the survival rate of patients [11, 12].

The results of this study showed that as of May 31, 2020, 13 of 86 breast cancer patients died. Among them, the mortality rate of the early recurrence group was 23.40% (11/47), which was higher than 5.13% (2/39) of the late recurrence group (*P* < 0.05). The median survival time of the early recurrence group was 26.8 months, which was lower than that of the late recurrence group of 54.3 months. Log-rank test *P*=0.012, the difference was statistically significant. The results showed that breast cancer recurrence time was correlated with survival prognosis, and patients with early recurrence had worse prognoses and higher mortality than patients with late recurrence. Studies have shown that surgical resection of the primary tumor will lead to the proliferation and recurrence of dormant cancer cells, resulting in poor prognosis for patients [13]. Compared with patients with late recurrence, patients with early recurrence have more irregular lesion morphology, stronger tumor heterogeneity, and more abundant blood flow, resulting in more aggressive recurrence of lesions, which is not conducive to the prognosis of patients. This is also the main reason for the significant difference in median survival time between the two groups in this study. DCE-MRI can predict the recurrence time of patients by showing the blood supply and tumor shape of the tumor, providing important reference value for clinical practice [14].

In conclusion, DCE-MRI images can clearly display the hemodynamic and morphological characteristics of tumor lesions, and have important value in predicting postoperative recurrence of breast cancer. Early recurrence of breast cancer has a worse prognosis, and DCE-MRI can predict postoperative recurrence time, providing an important reference for clinical practice. In addition, the shortcoming of this study is that the included samples were small, and the sample size could be expanded in the future to further verify the results of this study and the possible mechanism.

## Figures and Tables

**Figure 1:** Morphological features of phase 3 DCE-MRI in late recurrence group.

**Figure 2:** Morphological features of phase 3 DCE-MRI in early recurrence group.

**Figure 3:** ROC curve of DCE-MRI predicting breast cancer recurrence time.

**Figure 4:** The prognosis and survival curve of breast cancer patients with recurrence in different periods.

**Table 1:** Comparison of DCE-MRI features of breast cancer recurrence between two groups (*n*, %).

Indexes		Early recurrence group (*n* = 47)	Late recurrence group (*n* = 39)	*χ* ^2^ value	*P* value
BPE	None/Mild	27 (57.45)	24 (61.54)	0.148	0.701
	Moderate/significant	20 (42.55)	15 (38.46)		

Shape	Round/oval	9 (19.15)	3 (7.69)	2.497	0.287
	Lobulated	7 (14.89)	8 (20.52)		
	Irregular shape	31 (65.96)	28 (71.79)		

Edge of the lesion	Smooth	5 (10.64)	4 (10.26)	0.231	0.891
	Irregular	37 (78.72)	32 (82.05)		
	Starburst shape	5 (10.64)	3 (7.69)		

Intralesional enhancement	Ring reinforcement	18 (38.30)	10 (25.64)	1.555	0.212
	Acyclic reinforcement	29 (61.70)	29 (74.36)		

Whole breast vascular increase	Mild to moderate	20 (42.55)	25 (64.10)	3.968	0.046
	Severe	27 (57.45)	14 (35.90)		

Adjacent blood vessels	Yes	30 (63.83)	15 (38.46)	5.499	0.019
	No	17 (36.17)	24 (61.54)		

TIC	Enhanced type	9 (19.15)	8 (20.52)	0.079	0.961
	Platform type	17 (36.17)	13 (33.33)		
	Outflow type	21 (44.68)	18 (46.15)		

**Table 2:** Comparison of breast cancer recurrence and DCE-MRI hemodynamics between two groups (*n*, ±*s*).

Indexes	Early recurrence group (*n* = 47)	Late recurrence group (*n* = 39)	*t* value	*P* value
TTP (min)	1.94 ± 0.63	1.96 ± 0.65	0.144	0.886
Max Conc (mmol)	0.05 ± 0.02	0.04 ± 0.01	2.840	0.006
AUC (mmol·min)	0.26 ± 0.08	0.21 ± 0.04	3.550	0.001
Max Slope (mmol/min)	0.10 ± 0.02	0.07 ± 0.01	8.520	0.001
K^trans^ (ml/min)	1.28 ± 0.15	1.34 ± 0.18	1.686	0.095
K_ep_ (ml/min)	3.07 ± 0.22	3.08 ± 0.15	0.241	0.810
V_p_	0.41 ± 0.19	0.43 ± 0.17	0.509	0.612

**Table 3:** The predictive value of DCE-MRI for breast cancer recurrence.

Indexes	Area under the predicted value curve	Asymptotic 95% confidence interval		Best cutoff	Sensitivity (%)	Specificity(%)
		Lower limit	Upper limit			
Whole breast blood vessel increase	0.706	0.573	0.840	0.415	59.4	82.1
Adjacent blood vessels	0.761	0.757	0.948	0.581	68.8	89.3
Max Conc	0.822	0.713	0.931	0.554	87.5	67.9
AUC	0.796	0.675	0.916	0.485	80.6	67.9
Max Slope	0.891	0.812	0.969	0.520	80.6	71.4
Phase 3 morphological characteristic parameter sphericity	0.838	0.737	0.938	0.563	81.3	75.0
DCE-MRI	0.918	0.853	0.983	0.710	78.1	92.9

## Data Availability

The raw data supporting the conclusion of this article will be available by the authors without undue reservation.
